# Triptolide Attenuates Neuropathic Pain by Regulating Microglia Polarization through the CCL2/CCR2 Axis

**DOI:** 10.1155/2021/8985721

**Published:** 2021-10-14

**Authors:** Xubin Bao, Cai Chen, Liyong Yuan

**Affiliations:** ^1^Department of Anesthesiology, Fenghua District People's Hospital, Ningbo 315500, Zhejiang Province, China; ^2^Department of Anesthesiology, Ningbo No. 6 Hospital, Ningbo 315040, Zhejiang Province, China

## Abstract

Triptolide (T10) is a common anti-inflammatory and analgesic drug. However, the activation of microglia and elimination of the corresponding inflammatory response are new targets for the treatment of neuropathic pain. Chemokine CCL (CCL2) is a key mediator for activating microglia. In this study, the effects of triptolide on the activation and polarization of microglia cells and CCL2 and its corresponding receptor, chemokine receptor 2 (CCR2), were mainly discussed. Microglia were stimulated with 1 *μ*g/mL lipopolysaccharide (LPS) and pretreated with 10, 20, and 40 nM T10 and CCR2 antagonist (RS102895), respectively. The quantitative polymerase chain reaction (QPCR) and western blot results showed that T10 could obviously inhibit the upregulation of CCL2 and CCR2 induced by LPS stimulation in microglia cells, inhibit the fluorescence intensity of glial fibrillary acidic protein (GFAP) and inducible nitric oxide synthase (iNOS) antibody immunostaining in cells, and upregulate the fluorescence intensity of arginase 1 antibody in cells. The expression of interleukin-6 (IL-6), interleukin-1*β* (IL-1*β*), and tumor necrosis factor-*α* (TNF-*α*) was inhibited in a dose-dependent manner. RS102895 can significantly reverse the activation and M2 polarization of microglia pretreated with 40 nM T10 and weaken the anti-inflammatory effect of T10. The addition of CCL2 did not extremely affect the function of RS102895. T10 may inhibit microglia activation and M1 polarization by inhibiting the expression of CCL2 and CCR2, promoting M2 polarization, reducing the level of inflammatory factors in cells, and exerting its analgesic effect, which is worthy of clinical promotion as a drug for neuropathic pain.

## 1. Introduction

Neuropathic pain refers to the changes and confusion in the process of sensory nerve signals when entering the spinal cord and brain caused by lesions or diseases of the somatosensory system in the absence of nociceptive stimulation, as a result of the body's pathological adaptive response [1, 2]. Neuropathic pain can be divided into chronic pain with neurologic characteristics and specific neuropathic pain including trigeminal neuralgia, central neuralgia, and painful diabetic neuropathy, which affect the quality of life of 7%–10% of the general population seriously [3]. Besides, moderate and severe neuropathic pain leads to severe disability in most patients, which results in employment difficulties for patients and a heavy burden on the society and medical system [2, 3].

In the past, plastic changes and sensory responses of somatosensory neurons were the main research directions for rational treatment of pain after neuropathy injury, but in recent years, studies have found that glial cells may be the key cells of neuropathic pain. Under the pathological state of glial cells, they can release a large number of cytokines and chemokines. It forms a close interaction with neurons to regulate the transmission of pain [4, 5]. In particular, microglia, as the main macrophages and immune response cells in the central nervous system, is a necessary condition for synaptic changes and pain allergy after nerve injury [4–7]. Studies have found that the signal cascades and mediators in microglia cells can indirectly change the harmful signals between cells, thus creating therapeutic effects on the surrounding cells. Microglia cells have become a powerful target in the targeted therapy of neuropathic pain [4, 8].

Chemokines are a family of cytokines that can induce chemotaxis, which can guide cells expressing chemokine receptors to migrate to sites with high concentrations of local chemokine ligand, thus leading to inflammatory response [9]. The signal CCL2 and its receptor CCR2 axis are related to a variety of inflammatory and neurodegenerative diseases, which are expressed in neurons and glial cells, and can coordinate communication between neurons, microglia, and astrocytes. Plasma cells are considered a potential target for the treatment of neuropathic pain, atherosclerosis, and other diseases [10, 11].

Because of the problems of addiction and drug abuse in most drugs, neuropathic pain is difficult to be effectively treated, and the choice of drug treatment is still controversial. It is still the focus of clinical research to find a safe and effective analgesic drug [12]. Triptolide (T10) is a natural tricyclic diterpenoid product isolated from the traditional plant *Tripterygium wilfordii* with strong biological activities such as anti-inflammatory and antitumor [13, 14]. T10 has an important therapeutic potential in Alzheimer's disease and other central nervous system diseases; in addition, it has been reported that plant compounds such as T10 and curcumin have an effective preventive effect on neuropathic pain [15, 16]. However, its specific role in neuropathic pain is still unclear. Therefore, this study mainly explores the effect of T10 on activated microglia cells and its possible mechanism, in order to provide theoretical and experimental basis for the clinical use of T10.

## 2. Materials and Methods

### 2.1. Cell Culture

Human microglia cells were purchased from Wuhan Puno Sai Life Technology Co., Ltd. Human microglia cells were cultured in a constant temperature incubator with 5% CO_2_ at 37°C using the special complete medium provided by the company. 98% T10 (Aladdin, T107400) was dissolved in dimethyl sulphoxide, microglia were stimulated by 1 *μ*g/mL LPS (Sigma-Aldrich, L6529) for 24 h, and blank group was set as control. Cells were treated with no or with 10, 20, or 40 nM T10 half an hour before LPS stimulation. Microglia were pretreated with 5 M chemokine receptors 2 (CCR2) antagonist (RS102895) (Sigma-Aldrich, R1903) and 50 ng/mL chemokine CCL (CCL2) (Abcam, AB269211) for 1 h, followed by 40 nM T10 and subsequent LPS stimulation.

### 2.2. RT-qPCR

Total RNA in cells was lysed using Trizol (Solarbio, YZ-15596026), and then the first cDNA was performed using TransScript ® Two-Step RT-PCR SuperMix, which was amplified by PCR in a PCR instrument (Bio-Rad, iCycler iQ). Primer sequences are shown in Table 1, and their expression levels were detected by 2^−△△CT^ with GAPDH as the internal reference, △Ct(*n*) = Ct target gene (*n*)−Ct internal reference gene (*n*); △△CT(*n*) = △Ct(*n*)−△Ct(1).

### 2.3. Western Blot

After the cells were dissolved with RIPA lysate, the supernatant was collected, and the protein concentration was determined with BCA assay. After conventional electrophoresis with 1-%SDS-PAGE, the cells were transferred to PVDF membrane and sealed with 5% BSA (Sigma, A1933) for 2 h, and the corresponding primary antibodies, CCL2 (Cell Signaling Technology, 1 : 1000, 2027), CCR2 (Cell Signaling Technology, 1 : 1000, 12199), and GAPDH (Cell Signaling Technology, 1 : 1000, 12199) 5174), were incubated overnight at 4°C, washed with TBST, and incubated at room temperature for 2 h with the corresponding secondary antibody (Cell Signaling Technology, 5151), using an enhanced chemiluminescence kit (Beyotime Biotechnology, P0018 m) for exposure and development.

### 2.4. Immunofluorescence

The cells were fixed with 4% paraformaldehyde (GBCBIO, G0528) for 30 min, washed with PBS 3 times, and then sealed at room temperature for 1 h in 0.1% Triton X-100 (Roche, 10789704001) and 5% BSA. The cells were incubated overnight with rabbit anti-GFAP, iNOS, and arginase 1 (Abcam; ab33922, ab178945, and ab96183) at 4°C, and the second antibody (Abcam; ab150077 and ab7481) was colocalized with FITC-labeled Alexa Fluor 488 or Alexa Fluor 555 on the next day (AB150077 and AB7481). The cells were incubated at room temperature for 1 h, stained with DAPI (Sigma, D9542) for 10 min, washed with PBS 3 times, and photographed using a confocal microscope.

### 2.5. ELISA

The cell supernatant was collected, and the concentrations of interleukin-6 (IL-6), interleukin-1*β* (IL-1*β*), and tumor necrosis factor-*α* (TNF-*α*) (Abcam; AB178013, AB214025, and AB181421) in the cell supernatant were determined strictly according to the instructions of the kit. The expression was taken as pg/ml.

### 2.6. Statistical Methods

Independent sample *t*-test and one-way analysis of variance were performed using GraphPad Prism 8.0. The experimental data were repeated three times and represented as mean ± standard deviation. *P* < 0.05 was considered statistically significant.

## 3. Results

### 3.1. T10 Inhibited the Expression of CCl2 and CCR2 in LPS-Stimulated Microglia

After microglia were treated with 1 *μ*g/mL LPS for 24 h, QPCR detected the expressions of CCL2 mRNA and CCR2 mRNA in cells. Compared with the CON group, the expressions of CCL2 mRNA and CCR2 mRNA in microglia in the LPS group were significantly upregulated (*P* < 0.05, Figure 1(a)). Western Blot results also showed that LPS stimulation could upregulate the protein levels of CCL2 and CCR2 in microglia cells (*P* < 0.05, Figure 1(b)). Microglia were pretreated with different concentrations of T10 before adding the LPS, and the results showed that T10 could obviously inhibit the upregulated mRNA and protein expressions of CCL2 and CCR2 in microglia which is stimulated by LPS in a dose-dependent manner.

### 3.2. T10 Inhibited Activation and M1 Polarization in LPS-Stimulated Microglia

Fluorescence microscope observation showed that the expression of markers of microglial activation (GFAP) was obviously increased (Figure 2(a)), the expression of markers of M1 polarization (iNOS) was extremely increased, and the expression of markers of M2 polarization (arginase 1) was significantly decreased (Figure 2(b)). Thus, QPCR further validated microglial activation and increased M1 polarization markers. In addition, LPS-stimulated microglia were pretreated with different concentrations of T10 (*P* < 0.05; Figure 2(c)), and the results showed that, with the increase of T10 concentration, the fluorescence intensity of GFAP and iNOS in microglia cells decreased, while the fluorescence intensity of arginase 1 increased.

### 3.3. T10 Inhibited the Release of Inflammatory Cytokines in LPS-Stimulated Microglia

The level of inflammatory cytokines in microglia cells was detected by ELISA, and the results showed that LPS stimulation extremely increased the expression levels of IL-6, IL-1*β*, and TNF-*α* in cells. The addition of T10 pretreatment could significantly reduce the level of inflammatory cytokines in cells after LPS stimulation (*P* < 0.05), which indicated that T10 had anti-inflammatory effect on microglia after LPS stimulation. See details in Figure 3.

### 3.4. T10 Regulated Microglia Polarization through the CCl2/CCR2 Axis and Reduced the Release of Inflammatory Factors

In order to further analyze the effect of T10 on LPS-activated microglia and the function of CCl2 and CCR2 in them, microglia were pretreated with 5M RS102895 for 1 h and then treated with 40 nM T10 for half an hour. LPS are used to stimulate the microglia for 24 h. The addition of RS102895 obviously reversed the reduced activation and enhanced M2 polarization of microglia treated with 40NM T10, while the fluorescence intensity and mRNA expression in cells treated with CCl2 showed no significant changes (Figures 4(a)–4(c)). ELISA showed that RS102895 extremely weakened the anti-inflammatory effect of T10, while the addition of CCl2 did not improve this result (*P* < 0.05; Figure 4(d)), which suggested that T10 may inhibit microglia activation and M1 polarization by regulating the CCl2/CCR2 axis, promoting M2 polarization, and playing an anti-inflammatory role.

## 4. Discussion

Neuropathic pain is a chronic pain state that occurs after nerve injury and often involves abnormal excitability of the nervous system [17]. Microglia are resident macrophages that are widely distributed throughout the central nervous system. Some studies have pointed out that, after peripheral nerve injury, microglia cells, as the most sensitive sensors in encephalology, will undergo a complex activation process and become “activated” microglia cells, thereby releasing a large number of substances which are beneficial or harmful to the surrounding cells. Enhanced sensitivity of peripheral and heat stroke nociceptors would lead to the occurrence and persistence of neuropathic pain [6, 17–20].

If damage occurs, the microglia will quickly make a series of responses from the resting state to proinflammatory or anti-inflammatory, causing diseases and playing a protective role [21]. Among them, in the case of LPS, A*β*, neuroinflammation, and tissue injury, microglia will differentiate into the classic activated phenotype M1, which would release proinflammatory cytokines such as IL-6, IL-1*β*, and TNF-*α*, chemokines such as CCl2, and REDOX factors such as iNOS, which could help other immune cells enter the damaged area and trigger an inflammatory storm [8, 20–23]. When microglia turn to another alternative activation mode, M2, the cells will release IL-10, TNF-*β*, and other anti-inflammatory factors, promoting the phenotypic inactivation of inflammatory cells, producing arginase 1, leading to the reduction of injury-type NO, and promoting tissue regeneration and tissue homeostasis [8, 20–22, 24]. Activated microglia interacts with astrocytes, epithelial cells, and other cells to release inflammatory mediators, thus increasing the excitatory current in neuronal NMDA receptors, reducing the inhibitory current, or activating more microglia, further damaging the homeostasis of neurons and promoting the release of hyperalgesia and prostaglandin. It leads to neuropathic pain in the end [22, 25, 26].

As a main chemokine collected by monocytes in the brain after various nerve injuries, CCL2 is a key mediator of microglia activation in the state of neuropathic pain. Studies have shown that injection of CCL2 into the spinal cord of young mice can obviously activate microglia with neuropathic pain-like behavior, while inhibition of CCL2 expression significantly reduces neuropathic pain in young mice [25, 27–29]. Studies have pointed that CCL2 and its receptor CCR2 are expressed in both spinal dorsal horn neurons and glial cells in animal models of neuropathic pain, and CCL2/CCR2 signaling may be involved in the activation of glial cells in neuropathic pain model rats and trigger persistent neuropathic pain after peripheral nerve injury [30]. In addition, Wu et al. [31] also found that the CCL2/CCR2 signaling pathway enhances NMDA-mediated synaptic transmission in middle spine neurons, or knockdown and antagonism of CCR2 expression can significantly inhibit NMDA receptor-mediated current and alleviate neuropathic pain and depressive behavior.

It is an important means to target the activation and polarization of microglia in the central nervous system by interfering the CCl2/CCR2 signaling axis. Xu et al. [32] found in their studies that preinjection of CCR2 antagonist could significantly reduce the activation of microglia cells, M1 polarization, and release of inflammatory cytokines after surgery, reducing the injury and death of neurons. Besides, the application of CCR2 antagonist in neuropathic pain showed the same analgesic effect as the microglial cell inhibitor minocycline, which was closely related to the downregulation of CCL2 and CCR2 expressions in microglia cells [33]. Inhibition of CCL2/CCR2 signals can effectively inhibit glial cell activation and relieve neuropathic pain [34].

In this study, LPS-stimulated microglia cells were pretreated with different concentrations of T10, and the results showed that T10 could extremely downregulate the expression of CCL2 and CCR2, inhibit the activation and M1 polarization of microglia cells, promote M2 polarization, and reduce the expression levels of IL-6, IL-1*β*, and TNF-*α* in cells. Moreover, RS102895 reversed the activation inhibition effect of T10 on microglia cells and the addition of CCl2 had no obvious antagonistic effect on RS102895. It was suggested that T10 may play an anti-inflammatory role by inhibiting microglial activation and M1/M2 polarization mediated by CCl2/CCR2 signaling axis. T10 is a bioactive compound for the treatment of inflammatory diseases, which can regulate the release of a variety of inflammatory mediators and show excellent therapeutic effects in nephritis, endocrine diseases, and neurodegenerative diseases [35]. Studies have pointed that T10 can block cytokines and chemokines that were produced by LPS stimulation in a dose-dependent manner, thus showing a powerful immunosuppressive effect. T10 was also found to be effectively inhibited in brain inflammation to prevent LPS-induced microglial activation and subsequent excessive release of TNF-*α* and NO [36, 37]. This study also supported the results of our study that T10 may inhibit the polarization of microglia and reduce the release of inflammatory factors by regulating the expression of CCL2 and CCR2.

In conclusion, this study firstly found that T10 can downregulate the expressions of CCL2 and CCR2 in LPS-induced microglia cells, inhibit the activation of microglia cells, promote the polarization of microglia from M1 to M2, and reduce the level of inflammatory factors in cells. Antagonistic CCR2 can reverse the effect of T10 on microglia, which suggested that T10 may inhibit microglia activation and promote M2 polarization through the regulation of the CCl2/CCR2 axis, and T10 may be an effective drug for the treatment of neuropathic pain.

## Figures and Tables

**Figure 1:** T10 inhibited the expression of CCL2 and CCR2 in LPS-stimulated microglia. (a) QPCR detected the mRNA expressions of CCL2 and CCR2 in microglia cells. (b) Western blot detected the protein expression of CCL2 and CCR2 in microglia cells. *Note*. ^*∗*^Compared with the CON group without LPS, *P* < 0.05; ^#^vs. LPS group without T10, *P* < 0.05.

**Figure 2:** T10 inhibited activation and M1 polarization in LPS-stimulated microglia. Microglia cells were observed under a fluorescence microscope. (a) Antibody immunostaining of activation marker (GFAP), 200×. (b) Immunostaining of M1 polarization marker (iNOS) and M2 marker (arginase 1) antibodies, 200×. (c) The mRNA expressions of GFAP, iNOS, and arginase 1 in microglia cells were detected by QPCR. *Note*. ^*∗*^Compared with the CON group without LPS, *P* < 0.05; ^#^vs. LPS group without T10, *P* < 0.05.

**Figure 3:** T10 inhibited the release of inflammatory cytokines in LPS-stimulated microglia. The microglia cells were detected by ELISA. Expression level of (a) IL-6, (b) IL-1*β*, and (c) TNF-*α*. *Note*. ^*∗*^Compared with the CON group without LPS, *P* < 0.05; ^#^vs. LPS group without T10, *P* < 0.05.

**Figure 4:** T10 regulated microglia polarization through the CCl2/CCR2 axis and reduced the release of inflammatory cytokines. Microglia cells were observed under a fluorescence microscope. (a) The situation of antibody immunostaining of activation marker GFAP, 200×. (b) The situation of immunostaining of iNOS, the M1 polarization marker, and arginase 1, the M2 marker, 200×. (c) The mRNA expressions of GFAP, iNOS, and arginase 1 in microglia cells were detected by QPCR. (d) Expression of inflammatory cytokines IL-6, IL-1*β*, and TNF-*α* in cells was detected by ELISA. *Note*. ^*∗*^Compared with microglia stimulated by LPS after addition of 40 nM T10, *P* < 0.05.

**Table 1:** Primer sequence.

Genes	Forward (5′-3′)	Reverse (5′-3′)
CCL2	GATCTCAGTGCAGAGGCTCG	TTTGCTTGTCCAGGTGGTCC
CCR2	CCACATCTCGTTCTCGGTTTATC	CAGGGAGCACCGTAATCATAATC
GFAP	CTGCGGCTCGATCAACTCA	TCCAGCGACTCAATCTTCCTC
iNOS	CAGGGTGTTGCCCAAACTG	GGCTGCGTTCTTCTTTGCT
Arginase 1	CCCTGGGGAACACTACATTTTG	GCCAATTCCTAGTCTGTCCACTT
GAPDH	GACAGTCAGCCGCATCTTCT	GCGCCCAATACGACCAAATC

## Data Availability

The data used in this research can be obtained from the corresponding author.
